The article "Bioactive Natural Products against Systemic Arterial Hypertension: A Past 20-Year Systematic and Prospective Review" was published in 2022. Journal: Evid Based Complement Alternat Med.

# Bioactive Natural Products against Systemic Arterial Hypertension: A Past 20-Year Systematic and Prospective Review

**DOI:** 10.1155/2022/8499625

**Published:** 2022-06-20

**Authors:** Maisa Gomes da Silva, Sara Léa Fortes Barbosa, Diego Santos Silva, Isadora Basílio Meneses Bezerra, Érika Alves Bezerra, Angélica Gomes Coelho, Ilmara Cecília Pinheiro da Silva Morais, Luis Mário Rezende-Júnior, Iolanda Souza do Carmo, José de Sousa Lima-Neto, Simón Gabriel Comerma-Steffensen, Antônia Maria das Graças Lopes Citó, Daniel Dias Rufino Arcanjo

**Affiliations:** ^1^Department of Biophysics and Physiology, Federal University of Piaui, Teresina, Piaui, Brazil; ^2^Department of Chemistry, Federal University of Piaui, Teresina, Piaui, Brazil; ^3^Faculty of Pharmacy, Federal University of Piaui, Teresina, Piaui, Brazil; ^4^Pulmonary and Cardiovascular Pharmacology, Department of Biomedicine, Aarhus University, Aarhus, Denmark; ^5^Department of Biomedical Sciences/Animal Physiology, Veterinary Faculty, Central University of Venezuela, Maracay, Aragua, Venezuela

## Abstract

**Background:**

Systemic arterial hypertension is one of the most common cardiovascular risks, corresponding to 45% of deaths involving CVDs. The use of natural products, such as medicinal plants, belongs to a millennial part of human therapeutics history and has been employed as an alternative anti-hypertensive treatment.

**Objective:**

The present review aims to prospect some natural products already experimentally assayed against arterial hypertension through scientific virtual libraries and patent documents over the past 20 years. *Search strategy*. This is a systematic review of the adoption of the PRISMA protocol and a survey of the scientific literature that synthesizes the results from published articles between 2001 and 2020 concerning the use of medicinal plants in the management of hypertension, including which parts of the plant or organism are used, as well as the mechanisms of action underlying the anti-hypertensive effect. Furthermore, a technological prospection was also carried out in patent offices from different countries in order to check technologies based on natural products claimed for the treatment or prevention of hypertension. *Inclusion criteria*. Scientific articles where a natural product had been experimentally assayed for anti-hypertensive activity (part of plants, plant extracts, and products derived from other organisms) were included. *Data extraction and analysis*. The selected abstracts of the articles and patent documents were submitted to a rigorous reading process. Those articles and patents that were not related to anti-hypertensive effects and claimed potential applications were excluded from the search.

**Results:**

Eighty specimens of biological species that showed anti-hypertensive activity were recovered, with 01 representative from the kingdom Fungi and 02 from the kingdom Protista, with emphasis on the families Asteraceae and Lamiaceae, with 6 representatives each. Leaves and aerial parts were the most used parts of the plants for the extraction of anti-hypertensive products, with maceration being the most used extraction method. Regarding phytochemical analyses, the most described classes of biomolecules in the reviewed works were alkaloids, terpenes, coumarins, flavonoids, and peptides, with the reduction of oxidative stress and the release of NO among the mechanisms of action most involved in this process. Regarding the number of patent filings, China was the country that stood out as the main one, with 813 registrations.

**Conclusion:**

The anti-hypertensive activity of natural products is still little explored in Western countries. Besides, China and India have shown more results in this area than other countries, confirming the strong influence of traditional medicine in these countries.

## 1. Introduction

Arterial hypertension (AH) is a complex, multifactorial, and polygenic disease dependent on diet, demographic, and genetic factors, resulting from the imbalance of several systems, considered a public health problem and a risk factor for cardiovascular diseases (CVD), promoting heart failure, kidney failure, and stroke. Defined by blood pressure levels, AH is characterized by persistent and sustained elevation of blood pressure (BP), that is, systolic BP (SBP) greater than or equal to 140 mm·Hg and/or diastolic BP (DBP) greater than or equal to 90 mm·Hg [1].

CVDs are the leading cause of death, hospitalizations, and outpatient care worldwide, including in developing countries such as Brazil. In 2017, complete and revised data from DATASUS showed the occurrence of 1,312,663 deaths in total, with a percentage of 27.3% for CVD, with AH associated with 45% of these cardiac deaths [2, 3]. Recently, a study led by Imperial College London in collaboration with the World Health Organization (WHO) showed that the number of adults with hypertension between 30 and 79 years of age has increased from 650 million to 1.28 billion over the past 30 years, mainly in developing countries. The study revealed that the prevalence of AH decreased in high-income countries (Canada, Peru, and Switzerland), while in low-income countries (Dominican Republic, Jamaica, Paraguay, Hungary, and Poland), there was a significant increase. The factors involved in this increase would be the aging of the population and greater exposure to other risk factors [4]. Projections show that by 2030, 41.4% of US adults will have hypertension, an increase of 8.4% from 2012 estimates [5].

Determined by the product of cardiac output (CO) and peripheral vascular resistance (PVR), blood pressure is regulated by neural, renal, humoral, endothelial, and local control mechanisms of cardiovascular and renal functions. In this way, SAH can develop from abnormalities in any homeostatic control mechanisms of PVR and/or CD [6]. Thus, the pathophysiology of AH involves changes in its different mechanisms (baroreflex dysfunction, increased sympathetic activation, alterations in the renin-angiotensin-aldosterone system, increased NAD(P)H oxidase activity, oxidative stress, and endothelial dysfunction) [7], whose common trait is endothelial dysfunction, characterized by the low availability of nitric oxide (NO) and the consequent local imbalance between factors of relaxation and constriction of arterioles [8].

Classically, the treatment of AH consists of the use of anti-hypertensive therapy, which, associated or not with other methods, such as lifestyle modifications, can effectively reduce morbidity and mortality related to this condition [7]. This information becomes of great relevance for both the academic community and the scientific community, as a way of designing new intervention strategies, so that the individual with this disease can achieve greater success in its control and treatment. Thus, pharmacological and nonpharmacological measures protect against endothelial dysfunction by helping to preserve cardiovascular function through the reduction of oxidative stress and other mechanisms [9].  Figure 1 summarizes some physiological mechanisms towards therapeutic approaches that can be addressed.

Although more than 50% of existing medicines are synthesized from substances extracted from plants and herbs, the search for active ingredients present in plants, thus creating the first medicines with the characteristics that we know today, began only in the twentieth century—nineteenth century, according to historical records [10]. Among the drugs used in clinical practice whose origin comes from natural products, we can mention ephedrine (from *Ephedra sinica*), aspirin (from *Salix alba*), lovastatin (from *Monascus purpureus*), and reserpine (from *Rauwolfia serpentina*), for example [11].

Based on such knowledge, the objective of this study was to develop a systematic evaluation of the research carried out over the past 20 years on natural products with anti-hypertensive activity, extracting relevant information from scientific articles and patents.

## 2. Material and Methods

Through the adoption of the PRISMA protocol, a systematic review was carried out using scientific articles that addressed the anti-hypertensive activity of natural products. Following the guideline proposed by Sampaio and Mancini [12], the following question was formulated: “How many natural products have proven anti-hypertensive activity and been described in scientific articles published over the past 20 years?” Thus, a search was carried out in May 2020 in the main virtual libraries: Capes Periodical Portal, SciELO (Scientific Electronic Library Online), and portal BVS (Virtual Health Library), using the following terms: anti-hypertensive OR hypertension AND “natural product” OR “medicinal plant.” The articles should have been published between 2001 and 2020 and written in English, Portuguese, and Spanish. In the VHL Regional Portal, only articles with full text available were evaluated (Figure 2).

After cataloging, the reading of the abstract of the articles was performed by two researchers independently. Scientific articles in which a natural product had been experimentally tested for anti-hypertensive activity (parts of plants, plant extracts, and products derived from other organisms) were accepted and articles that were not intended to evaluate the anti-hypertensive function, and those related to synthetic or semisynthetic products were excluded. Subsequently, information was extracted on the species used (family, chemical constituents, and mechanisms of action) for the construction of the work.

Concomitantly, a prospective technological study was carried out in order to verify the patents deposited and published over the past 20 years, in order to obtain a current view related to the technologies used for medicinal plants in the prevention of hypertension. A search was carried out from databases associated with the INPI (National Institute of Industrial Property), the USPTO (United States Patent and Trademark Office), the EPO (European Patent Office), the WIPO (World Intellectual Property Organization), and the LATIPAT, using the keywords: medicinal plant (s) and herb(s) associated with the words hypertension, anti-hypertensive, and hypotensive activity. In the case of duplication, the patent of the database other than WIPO was recorded. After an exploratory reading of the titles and abstracts, those that were in accordance with the objective of the study were selected and fully analyzed.

## 3. Results and Discussion

The search for the terms associated with hypertension, anti-hypertensive drugs, natural products, and medicinal plants in three selected virtual libraries yielded a total of 219,519 scientific articles published between the years 2001 and 2020. Of this total, 3,813 came from the search on the Capes Periodicals Portal, 3,203 from SciELO and 212, 503 from the VHL portal. Ninety-five articles were selected after applying the inclusion and exclusion criteria. Within these works, 80 specimens of biological species that showed anti-hypertensive activity were identified, with 01 representative of the Fungi kingdom and 02 of the Protista kingdom (Table 1). Species from the most different families were found, especially the Asteraceae and Lamiaceae families, with 6 representatives each (Figure 3).

The Asteraceae family is one of the largest of the angiosperms group, with about 180 genera, being considered one of the most important sources of plant species of therapeutic interest [13]. In Brazil, it covers the phytogeographic domains of the Caatinga, Amazon, Pantanal, Pampa, Atlantic Forest, and Cerrado [14]. It bears great importance for the composition of the vegetation of different places, being one of the richest families [15]. Its plants can produce a wide variety of secondary compounds; the most common compounds are phenolic acids, polyacetylenes, flavonoids, coumarins, benzofurans, and terpenoids such as monoterpenes, diterpenes, triterpenes, sesquiterpenes, and especially sesquiterpene lactones [16].

In turn, the Lamiaceae family, with 295 genera and about 7,775 species, another great representative of angiosperms [17], is a group with a cosmopolitan distribution, occurring mainly in open savannas and mountainous regions with a tropical to subtropical climate [18]. Being represented in Brazil by 34 genera and 498 species, the species of this family produce a wide variety of secondary metabolites [19] and accumulate substances with great structural diversity, such as steroids, flavonoids, iridoids, and terpenoids, including triterpenes. The latter are known to have anti-tumor, anti-HIV, anti-inflammatory, anti-oxidant, anti-bacterial, and anti-fungal activities, among others [20]. Thus, other members of these families deserve to be studied.

Popular observations on the use and effectiveness of medicinal plants significantly contribute to the dissemination of the therapeutic virtues of plants, frequently prescribed, for the medicinal effects they produce, despite not having their known chemical constituents. Indirectly, this type of medicinal culture draws the interest of researchers in studies involving multidisciplinary areas, such as botany, pharmacology, and phytochemistry, which together enrich the knowledge about the world flora [21].

In general, the choice of a particular medicinal plant is made through the ethnopharmacological approach. Once the plant species to be studied is defined, the place of the collection is also defined, as well as the part of the plant that will be investigated (root, stem bark, stem, branches, leaves, flowers, and fruits) for carrying out the phytochemical study. Thus, in a project that links phytochemistry with pharmacology, the part of the plant that is used in folk medicine should be chosen for collection [21]. During the survey, it was observed that the leaves and aerial parts, roots, and seeds were the most used parts of the plants for the extraction of anti-hypertensive products, as shown in Figure 4(a).

The search for bioactive compounds of natural origin has increased considerably over the past two decades, mainly due to their preventive potential and in the treatment of cardiovascular, chronic, and neurodegenerative diseases [22]. In this sense, finding efficient extractive methods as well as the characterization of bioactive compounds from natural sources is a great challenge for researchers. Extractive methods for obtaining plant extracts include maceration, infusion, percolation, decoction, continuous hot extraction (Soxhlet), countercurrent extraction, microwave-assisted extraction, ultrasound, supercritical fluid, and turbolysis. In addition to the extractive methods, there are several factors that influence the extraction, such as the part of the plant material used, its origin, the degree of processing, the particle size, the solvent used, the extraction time, temperature, polarity, solvent concentration [23], and how communities do it [24]. Maceration was the most used extraction method in the research reviewed, followed by infusion/decoction and parallel Soxhlet. Other techniques such as percolation and critical superfluid extraction occurred less frequently (Figure 4(b)).

In order to quantify and qualify the chemical constituents of plant extracts, whose beneficial effects of some substances of certain species act as a key factor for the development of research bases for future applications of these bioactives [25], a preliminary phytochemical investigation is carried out to recognize the chemical constituents and/or assess their presence in the species being studied [26]. Specifically, phytochemical screening makes it possible to carry out preliminary tests to identify the presence of chemical compounds in certain plant species and thus link them to possible biological activities.

For example, alkaloids have anti-bacterial, anti-fungal, anti-plasmodic, and anti-tumor properties [27, 28] due to the ability to destabilize biological membranes. They also have the ability to inhibit the synthesis of DNA and RNA by binding to nucleic acids and intercalating into the double helix [29]. Examples of alkaloids currently used are morphine (analgesics), scopolamine (anti-cholinergics), theophylline (diuretics), vincristine (anti-tumours), and codeine (anti-tussives) [30].

Flavonoids are the most numerous compounds in angiosperms and have anti-inflammatory, anti-allergic, anti-ulcerogenic, anti-viral, anti-proliferative, anti-oxidant, hepatoprotective, anti-thrombic, and anti-carcinogenic activities [29, 30]. Tannins are phenolic compounds that have the property of complexing with metal ions and macromolecules such as proteins and polysaccharides, so they play the role of anti-oxidant and protector against herbivores and microorganisms. They are used as anti-septics, astringents, anti-diarrheals, wound healing, burns, and inflammation due to their ability to precipitate proteins [29–31]. They also have the ability to stimulate phagocytic cells [30].

Terpenes make up some essential oils and, therefore, act to attract pollinators. They also have insecticidal, anti-microbial, hepatoprotective, analgesic, anti-inflammatory, anti-microbial, and hemolytic action, among others [29, 31]. Triterpenes have anti-inflammatory, analgesic, cardiovascular, and anti-tumor effects [32].

Saponins have the ability to decrease the surface tension of water and, *in vitro*, cause erythrocyte hemolysis. They alter membrane permeability by lipophilic action and complexation with lipids and cell membrane proteins, which causes cell destruction. Therefore, they have toxic characteristics [31]. They also perform molluscicidal, anti-fungal, anti-microbial, anti-parasitic, anti-viral, cytotoxic, and anti-tumor functions [30].

Phenolic compounds have the ability to neutralize free radicals, inhibiting the risk of cardiovascular disease, diabetes, tumors, and inflammatory processes. Coumarins are used for dermatoses, psoriasis, vitiligo, and other skin diseases; they are also anti-coagulants and laxatives, such as anthraquinones. Catechins are anti-oxidants, thermogenic, anti-inflammatory, and anti-carcinogenic. Steroids have cardiotonic functions, activators of anabolism, precursors of vitamin D, and contraceptives [30].

Regarding phytochemical analyses, the most described classes of biomolecules in the reviewed works were alkaloids, terpenes, coumarins, flavonoids, and peptides (Table 1). Thus, when relating them to anti-hypertensive activity, the focus of the prospective studies, we observed that alkaloids, such as reserpine and alstonine, reduce the availability of norepinephrine and, therefore, act as vasodilators. Flavonoids such as quercetin and rutin are primarily active in the myocardium and reduce cardiac output. Linoleic acid inhibits atherosclerosis-generating deposits of cholesterol and triglycerides [109]. Phenolic compounds are anti-oxidants responsible for scavenging free radicals, capable of minimizing the harmful effects of ROS, and considered potential for the prevention of cardiovascular diseases [36].

The control of BP is made through two main mechanisms: neural and humoral. The neural mechanism is made by the autonomic nervous system composed of the sympathetic and parasympathetic systems, which act by increasing or decreasing heart rate as well as acting on peripheral vascular resistance. Humoral control is carried out by several substances that directly interfere with peripheral vascular resistance. Thus, the increase in vasodilating substances such as NO can contribute to an improvement in SAH. On the other hand, the renin-angiotensin system (RAS) plays a fundamental role due to its vasoconstrictor action, mainly through angiotensin II (Ang II) [110].

The classic view of the RAS is given by the production of angiotensinogen by the liver, being released into the circulation, where it is found in high concentrations. In the circulation, angiotensinogen undergoes the action of renin, a glycoproteolytic enzyme of renal origin [111]. After being synthesized and released into circulation, renin promotes the conversion of angiotensinogen into Angiotensin I (Ang I) [112], and this is converted into angiotensin II (Ang II) by the catalytic action of angiotensin-converting enzyme (ACE) [113]. This conversion occurs almost exclusively in the vessels of the lungs, catalyzed by the ACE present in the endothelium of the pulmonary vessels.

The effects of Ang II are mediated by two distinct types of receptors: AT_1_ and AT_2_, and the greatest interaction of this peptide occurs via the AT_1_ receptors, causing vasoconstrictor action, arrhythmogenic effect, cell proliferation, thrombosis, coagulation, inflammation, and hypertrophy of vascular smooth muscle [114, 115]. This Ang II signaling pathway with AT_1_ receptors is carried out by the activation of the *G* protein, with consequent activation of phospholipase C-*β* and formation of 1,4,5-triphosphate and diacylglycerol, which in turn increases the intracellular concentration of calcium leading to vasoconstriction [116]. In addition to these effects, it is known that *q* Ang II via AT_1_ receptors stimulates aldosterone secretion by the zona glomerulosa of the adrenal cortex [117]. Contrary to this, the interaction of Ang II with the AT_2_ receptor has an antagonistic effect on the action of the Ang II axis–AT_1_ receptor, resulting in the formation of NO, and consequent vasodilation [118].

In addition to the physiological effects of controlling cardiovascular function, Ang II is also involved in the pathophysiology of cardiovascular diseases since this peptide induces the formation of reactive oxygen species (ROS) in the endothelium and vascular smooth muscle [119]. This process occurs via AT_1_ receptors and consequent activation of the enzyme NAD (P) H oxidase [120], which reduces the oxygen molecule, forming O_2_^−^. The latter is dismutated to H_2_O_2_ by the action of the enzyme superoxide dismutase (SOD) or reacts with NO to form peroxynitrite (ONOO^−^) mainly under pathophysiological conditions [121].

The lower availability of NO favors greater activity of endothelin-1 (ET-1) or endothelium-derived contracting factor (EDCF) promotes endothelial cell growth and vasoconstriction and, therefore, participates in the pathogenesis of oxidative stress of SAH [122, 123]. Thus, vascular oxidative stress would result in SAH, since vasoconstrictor factors would be in preponderance in relation to vasodilator factors.

NO biosynthesis comprises one of the most important functions of L-arginine metabolism in the body. NO is formed from the terminal nitrogen of guanidine present in L-arginine, under the catalytic action of the enzyme nitric oxide synthase (eNOS), generating equimolar concentrations of L-citrulline and NO [124]. Once released, NO rapidly diffuses from the generating cell (endothelial cells) to the target cell (smooth muscle of the blood vessel), where it interacts with the heme group of soluble guanylate cyclase (GCs) stimulating its catalytic activity, leading to the formation of cGMP, which in turn decreases intracellular calcium (Ca^2+^) levels, reducing vascular tone. The mechanisms by which the NO/cGMP pathway induces vasodilation include inhibition of inositol-1,4,5-triphosphate (IP3) generation, increased cytosolic Ca^2+^ sequestration, myosin light chain dephosphorylation, inhibition of Ca^2+^ influx, activation of protein kinase, stimulation of membrane Ca^2+^ ATPase, and opening of K^+^ channels [125].

Regarding the mechanisms of action used in research cataloged to support the anti-hypertensive effect of the species evaluated, NO release, reduction of oxidative stress, ACE inhibition, Ca^2+^ channel block, RAAS modulation, activation of K^+^ channels, inhibition of nuclear kappa transcription factor (NF-*κ*B), and increase in natriuresis can be observed (Figure 5). Among the possible study models, the research was carried out in *in vivo*, *ex vivo*, *in vitro*, and *in silico* studies, including studies in humans (Table 1).

As for the number of patents deposited in the databases according to the keywords used, it was observed that the WIPO database markedly recovered 925 documents, followed by the EPO and USPTO, with only 6 and 2 documents, respectively. In the others, INPI and LATIPAT, no patents were found. This may suggest a lack of interest on the part of research centers or industries to innovate in anti-hypertensive products, even though hypertension is one of the main causes of death in the world and 25% of currently available drugs originate from medicinal plants [126].

China was the country with the highest number of patent filings with 813 registrations. The other countries and their respective patent offices showed very low values when compared to China: the Republic of Korea with 75, the United Kingdom with 15, the World Intellectual Property Organization with 12, the European Patent Office with 7, Japan with 6, the United States with 2, and Canada, Russia, and France with 1 each (Figure 6). Although Brazil is a country rich in biodiversity and one that develops a lot of research on medicinal plants, research in the patent databases revealed a lack of interest in the development of technologies with market potential related to anti-hypertensive herbal medicines.

The superiority in the number of patents filed by China is related to the economic and technological position of this country in relation to the world scenario, as China has been increasingly establishing itself as a producer of knowledge and technological development, mainly through the work of pharmaceutical multinationals, electronics, and food, as well as the implementation of scholarship programs to encourage research. At the same time, traditional Chinese medicine is accompanied by a vast agricultural experience, which favors the study and development of technological alternatives that take advantage of the therapeutic potential of different plant species, especially regarding such promising applicability, for example, prevention and treatment of hypertension [127].

As for the temporal evolution of the number of patent filings (Figure 7), the sharp increase in the years 2014 and 2015 is noticeable. Regarding this increase, it is important to mention that in 2010 in the National Patent Development Strategy in China, the government defined benchmarks for future performance by 2015, setting the number of patent applications to reach two million, which would quadruple the number of applications in 2010, so that by 2015, China would be among the top two countries in a number of invention patents granted to national applicants. Such targets may have greatly influenced the significant increase in the number of patents registered in 2014 and 2015 [128].

## 4. Conclusion

From this perspective, the anti-hypertensive activity of natural products is still little explored, especially in Western countries. In this sense, China and India have shown more results in this area than other countries, confirming the strong influence of traditional medicine in these countries. Leaves and aerial parts were the main fractions of plants with potential exploitation. The maceration technique was the most used in obtaining the extract. The Fabaceae family was the most cited, which may indicate that more plant species belonging to this family should be studied regarding the anti-hypertensive potential. The largest number of patents related to anti-hypertensive herbs is deposited in WIPO. China is the country that invests most in research with the technological development of products from medicinal plants for the treatment and prevention of hypertension. This study was able to provide theoretical subsidies for future research with medicinal plants on the use of natural products as a coadjuvant in the treatment of systemic arterial hypertension.

## Figures and Tables

**Figure 1:** Main mechanisms and signaling pathways involved in blood pressure control.

**Figure 2:** Process of the research and treatment protocol of scientific production articles about natural products that possess anti-hypertensive activity.

**Figure 3:** Distribution of the main families used in scientific research on natural products with anti-hypertensive activity published in the virtual libraries portal BVS, CAPES, and SciELO from 2001 to 2020.

**Figure 4:** Percentages of the main chosen plant parts (a) and the main extractive methods (b) used to obtain the different natural products with anti-hypertensive activity retrieved from the virtual libraries BVS, CAPES, and SciELO over the period between 2001 and 2020.

**Figure 5:** Distribution of the anti-hypertensive mechanisms elucidated in the scientific research of natural products with anti-hypertensive activity published in the virtual libraries BVS Portal, CAPES, and SciELO in the period of 2001 to 2020.

**Figure 6:** Distribution of patents deposited in accordance with the depositary office in the INPI (National Institute of Industrial Property, Brazil), the USPTO (European Patent Office), the EPO (European Patent Office), the WIPO (World Intellectual Property Organization), and the LATIPAT.

**Figure 7:** Patent deposit evolution over the past 20 years on the bases of the INPI (National Institute of Industrial Property, Brazil), the USPTO (United States Patent and Trademark Office), the EPO (European Patent Office), the WIPO (World Intellectual Property Organization), and the LATIPAT.

**Table 1:** Chemical constituents related to the anti-hypertensive effect of the species, mechanisms of action, study model used, and other relevant information in the publications of 2001–2020.

Species	Family	Used part (s)	Chemical constituents/classification	Mechanisms of action	Study model	Reference
*Agelanthus dodoneifolius*	Loranthaceae	No data	Dodonein (lactone)	Blockade of the L-type calcium channels and inhibition of carbonic anhydrase in smooth muscle cells	*Ex vivo* assays for vasodilation in rat aortic rings; *in vitro* assay by the culture of vascular smooth muscle cells and determination of messenger RNA of carbonic anhydrase isozyme A in smooth muscle cells	[33]
*Allium cepa*	Amaryllidaceae	Rhizome	Diallyl thiosulphinate, methyl allyl thiosulphinate, allylmethyl thiosulphinate, protocatechuic acid, vanillic acid, p-hydroxybenzoic acid, ferulic acid, protocatechuic acid, vanillic acid, p-hydroxybenzoic acid, *ferulic* acid, and sinapinic acid	Inhibition of angiotensin-converting enzyme	*In vitro* angiotensin-converting enzyme inhibitory assay	[34]
*Allium sativum*	Amaryllidaceae	Rhizome	S-allyl cysteine	Inhibition of angiotensin-converting enzyme	*In vivo* assays with mice with fructose-induced hypertension	[35]
*Alpinia zerumbet*	Zingiberaceae	Leaves	Routine and kaempferol-3-O-*β*-D-glucuronide (flavonoids)	Stimulates NO/cGMP pathway	*Ex vivo* tests of isolation of the superior mesenteric artery of rats	[36]
*Annona muricate*	Annonaceae	Leaves	Roseoside, isolariciresinol 9-O-*β*-D-xyloside, massonianoside B, icariside E4, and nicotiflorin	Anti-oxidant, anti-inflammatory, and anti-vascular remodeling properties and reduced AT1 receptor expression	*In vitro* assay in angiotensin II (Ang II) stimulated H9C2 cells	[37]
*Angelica dahurica*	Apiaceae	Root	Imperatorin	Reduction of oxidative stress and prevention of hypertension-related renal injury	*In vivo* assay in rats with renovascular hypertension and *ex vivo* assays that evaluate the cellular redox state	[38]
*Angelica decursiva*	Apiaceae	Root	Decursin and nodakenin	Opening of the potassium channels	Assays in rat aortic arteries	[39]
*Apium graveolens*	Apiaceae	Seed	3-n-butylphthalide	Reduction of renal fibrosis; reduction of oxidative stress; decreased levels of TNF-*α*, IL-6, and NF-*κ*B	*In vivo* assays with spontaneously hypertensive rats	[40]
*Arbutus andrachne*	Ericaceae	Root, leaves, and fruit	Phenols, flavonoids, tannins, and anthocyanins	Reduction of oxidative stress	*Ex vivo* tests for vasodilation in rat aorta rings with intact endothelium; *ex vivo* assays that evaluate the cellular redox state	[41]
*Arbutus unedo*	Ericaceae	Root	Tannins and flavonoid (quercetin and tannic acid)	Stimulation of the endothelial nitric oxide synthase and activation of muscarinic receptors	*Ex vivo* tests for vasodilation in rat aorta rings with intact endothelium	[42]
*Azadirachta indica*	Meliaceae	Leaves	No data	Activation of muscarinic receptors in the heart, reducing the heart rate and increasing peripheral resistance	*In vivo* assay in rats with hypertension induced by DOCA-salt injection	[43]
*Berberis vulgaris*	Berberidaceae	Fruit	No data	Activation of the l-arginine-nitric oxide pathway	*In vivo* assay in rats with hypertension induced by DOCA-salt injection, *in vitro* studies in aortic rings, and *in vitro* studies in the isolated perfused mesenteric beds	[44]
*Bidens pilosa*	Asteraceae	Leaves	Alkaloids, saponins, flavonoids, polyacetylenes and triterpenes, phenylheptatriyne, linoleic acid, and linolic acid	Blocking of calcium channels	*Ex vivo* assays for vasodilation in rat aortic rings	[45]
*Boerhavia diffusa*	Nyctaginaceae	Root	Culubin (diterpenoid)	Blocking of calcium channels	*In vivo* assay in rats with hypertension caused by obesity induced by a lipid-rich diet	[46]
*Cassia tora*	Fabaceae	*Seed*	Chrysofanol, Aurantium Obtusine, alaternine, and chrysobthysin (anthraquinones)	Inhibition of angiotensin-converting enzyme	*In vitro* assays	[47]
*Cecropia pachystachya*	Urticaceae	Leaves	Ambaina and ambainina, long-chain carboxilic acids, and *β*-sitosterol	Sympathic blockade in vessels and tachycardia by vagal inhibition in the heart	*In vivo* assay in normotensive Wistar rats through cannulation of internal carotid artery	[48]
*Cleistanthus collinus*	Phyllanthaceae	Leaves	Cleistantin A and B (glycosides)	Inhibition of angiotensin-converting enzyme	*In silico* molecular interaction	[49]
*Crataegus tanacetifolia*	Rosaceae	Leaves	Hyperoside	Increase in kidney NOS activity, diuretic activity, and efflux of water and sodium, preventing hyperlipidemia and decrease in body weight	*In vivo* assay in normal male Wistar albino and L-NAME-induced hypertensive rats	[50]
*Codonopsis lanceolata*	Campanulaceae	Rhizome	Lancemaside A	Increase in NO levels by eNOS (inducible NO synthase)	*In vitro* assay in human umbilical vein endothelial cells	[51]
*Coffea*	Rubiaceae	Fruit	Chlorogenic acids	Stimulation of the endothelial nitric oxide synthase	A double-blind, randomized, placebo-controlled study in humans	[52]
*Coix larchryma-jobi*	Poaceae	Seed	Glutelin hydrolyzate	Inhibition of angiotensin-converting enzyme	*In vivo* assays in hypertensive rats	[53]
*Cordyceps sinensis* ^*∗*^	Clavicipitaceae	Entire organism	Mannose, glucose, and galactose (polysaccharide fraction)	Increase in NO levels and decrease of the levels of endothelin-1, epinephrine, noradrenaline, angiotensin II, and TGF-*β*1	*In vivo* assays with spontaneously hypertensive rats	[54]
*Coriandrum sativum*	Apiaceae	Fruit	Camphor, camphene, carvone, cineole, cimene, coriandrine, limonene, linoleic acid, myrcene, myristic acid, oleic acid, palmitic acid, *α*-phenyltriene, *β*-phenylandrene, and *α*-terpinene, among others	Blockade of calcium channels, interaction with muscarinic receptors and diuretic effect	*In vivo* assays in normotensive mice and *ex vivo* assays in isolated tissue preparations	[55]
*Crocus sativus*	Iridaceae	Flower	Crocin, crocetina, and Safranal	Release of nitric oxide, reduction of oxidative stress, and modulation of the renin-angiotensin system	*In vivo* assay in rats through cannulation of arteries and femoral veins of rats with hypertension induced by Ang-II	[56]
*Croton schiedeanus*	Euphorbiaceae	Aerial parts (stem and leaves)	Flavonoids, diterpenoids, and phenylbutanoids	Stimulation of NO/cGMP pathway	*In vivo* assays in mice with hypertension by chronic inhibition of nitric oxide and *ex vivo* assay in isolated tissue preparations	[9]
*Cucurbita pepo*	Cucurbitaceae	Seed	Cucurbitacins (triterpenes); lutein, carotene, and beta carotene(carotenoids); unsaturated linoleic and oleic acids	Increase of NO levels	*In vivo* assays in mice with chronic inhibition of nitric oxide and *in vitro* assays	[57]
*Curcuma spp.*	Zingiberaceae	Rhizome	Curcumin, demethoxycurcumin, and bisdemethoxycurcumin	Blocking of calcium channels and the partial inhibition of b-adrenergic receptors	*Ex vivo* vasodilation assay on intact endothelium pigs basilar arteries pre-contracted	[58]
*Cyclocarya paliurus*	Juglandaceae	Leaves and seeds	Polysaccharides	Reduction of oxidative stress	*In vitro* and *in vivo* assays using hypertensive rats	[59]
*Dendranthema indicum*	Asteraceae	Flower	Linarin	Modulation of the Renin-angiotensin system	*In vivo* assays with spontaneously hypertensive rats	[60]
*Dicksonia sellowiana*	Dicksoniaceae	Leaves	Polyphenols	Reduction of oxidative stress, activation of the pathway PI3K/Akt/eNOS	*Ex vivo* tests on isolated tissues; *in vitro* assay on pig endothelial cell culture; *in vivo* tests with spontaneously hypertensive rats	[61]
*Dioscorea opposita*	Dioscoreaceae	Rhizome	Saponins, starch, mucopolysaccharides, protein, amino acids, mucilage, and polyphenols	Inhibition of angiotensin II converting enzyme, inhibition of endothelin-1 and reduction of oxidative stress	*In vivo* assay in rats with renovascular hypertension and *ex vivo* assays that evaluate the cellular redox state	[62]
*Eclipta alba*	Asteraceae	Aerial parts	Culubin (diterpenoid)	Diuresis due to increase in sodium excretion	*In vivo* assay in rats with hypertension caused by obesity induced by a lipid-rich diet	[46]
*Eucommia ulmoides*	Eucommiaceae	Stem bark	Wogonin (flavonoid)	Inhibition of the intracellular release of Ca^2+^ and the extracellular influx of Ca^2+^	*Ex vivo* testing on isolated tissue preparations	[63]
*Ficus deltoidea*	Moraceae	Leaves	*β*-amyrin, lupeol, *β*-amyrin cinnamate and bergapten, tanacetene, *β*-elemene, stigmasterol, *β*-sitosterol, lupenone, and *α*,*β*-amyrenone, as well as alkaloids, saponin, phenols, flavonoids, and tannins	Modulation of the renin-angiotensin-aldosterone system, anti-oxidant and endothelial system	*In vivo* assays with spontaneously hypertensive rats	[64]
*Gardenia jasminoides*	Rubiaceae	Fruit	Crocetin (carotenoid)	Increase in NO levels by eNOS and iNOS (inducible NO synthase)	*In vivo* assays with spontaneously hypertensive rats, *ex vivo* vasodilation assay on intact endothelium mouse aorta rings, and *in vitro* assays	[65]
*Glycine Max*	Fabaceae	Seed	Equol (flavonoid)	Diuresis by an increase in sodium excretion and increases transcription of the enzyme eNOS	A double-blind, randomized, placebo-controlled study in humans	[66]
*Gomphrena celosioides*	Amaranthaceae	Aerial parts	Phenolic acids and flavonoids	Increased levels of bradykinin, prostaglandins, and NO	*In vivo* assays in hypertensive animals	[67]
*Hibiscus sabdariffa*	*Malvaceae*	Flower	Anthocyanins	Increase in NO by activation of PI3K/Akt/eNOS pathway and activation of potassium channels	*Ex vivo* rat assays in isolated tissue preparations	[68]
*Inula viscosa*	*Asteraceae*	Leaves	Phenolic compounds and flavonoids	Inhibition of angiotensin-converting enzyme	*In vivo* assays in hypertensive adult rats	[69]
*Leersia hexandra*	Poaceae	Aerial parts	Not identified	Anti-oxidative and lipid-lowering effect	*In vivo* assays with hypertensive rats induced by oral administration of ethanol	[70]
*Lippia origanoides*	Verbenaceae	Aerial parts	Naringenin and pinocembrina (flavonoids), quercetin (flavonol), and luteolin (flavones)	Activation of calcium-activated potassium channels and increase in cAMP and and cytosolic cGMP	*In vivo* assays in mice with hypertension by chronic inhibition of nitric oxide	[71]
*Lithocarpus polystachys*	Fagaceae	Leaves	florizine, fluoxetine, quercetin, dihydrochalcone-20-b-D-glucopyranoside, luteolin, and quercetin (Flavonoids)	Modulation of the renin-angiotensin-aldosterone system and reduction of oxidative stress	*In vivo* assays with spontaneously hypertensive rats and normotensive rats; *in vitro* assays	[72]
*Lonchocarpus xuul*	Fabaceae	Root	Dihydrospinochalcone-A and isocordoin	Activation of potassium channels and activation of NO/sCG/PKG pathway	*In vivo* assay in spontaneously hypertensive rats; *ex vivo* testing on isolated tissue preparations; molecular interaction *in silico*	[73]
*Lycopersicon esculentum*	Solanaceas	Fruit	*α*-tocopherol and the carotenoids: lycopene, *β*-carotene, phytoene, and phytofluene	Attenuation of inflammatory signaling by the inhibition of the NF-*k*B transcription factor in endothelial cells	A double-blind, randomized, placebo-controlled study in humans; *in vitro* assay on human endothelial cell culture	[74]
*Mentha x villosa*	Lamiaceae	Leaves	No data	Active vascular relaxation	*In vivo* assay in rats with hypertension induced by DOCA-salt injection	[75]
*Mesona procumbens*	Lamiaceae	Leaves	Caffeic acid (polyphenol)	Reduction of oxidative stress	*In vivo* assay in spontaneously hypertensive rats and *ex vivo* assay evaluating the cellular redox state	[63]
*Mimosa caesalpiniifolia*	Fabaceae	Inflorescences	Gallic acid, rutin, quercetin, and vicenine (flavonoids)	Activation of the muscarinic and ganglionic pathways and blockade of the transmembrane calcium influx	*In vivo* assay in normotensive mice; *ex vivo* testing on isolated tissue preparations	[76]
*Mitragyna ciliata*	Rubiaceae	Stem Bark	Alkaloids (mitragynine, mitraphylline, and rhynophylline) and/or flavonoid	Blocking of calcium channels	*Ex vivo* rat assays in guinea pig and rat isolated aortic rings	[77]
*Mixture containing Pine densiflora,*	Pinaceae	Leaves	Roseoside, isolariciresinol 9-O-*β*-D-xyloside, massonianoside B, icariside E4, and nicotiflorin	Anti-oxidant, anti-inflammatory, and anti-vascular remodeling properties and reduced AT1 receptor expression	*In vitro* assay in Angiotensin II (Ang II)-stimulated H9C2 cells	[37]
*Momordica charantia*	*Cucurbitaceae*	Leaves	Roseoside, isolariciresinol 9-O-*β*-D-xyloside, massonianoside B, icariside E4, and nicotiflorin	Anti-oxidant, anti-inflammatory, and anti-vascular remodeling properties and reduced AT1 receptor expression	*In vitro* assay in Angiotensin II (Ang II) stimulated H9C2 cells	[37]
*Morinda citrifolia*	*Rubiaceae*	Root	Alkaloids, phenolic compounds, sterols, flavonoids, tannins, coumarins, and anthraquinones	Blocking of calcium channels and release of intracellular calcium	*Ex vivo* rat assays in tissue preparations isolated from rats	[78]
*Moringa oleifera*	Moringaceae	Leaves	Nitrile, glucosinolates and thiocarbamate glycosides, flavonoids, phenolic acids, tannins, quercetin-3-O-glucoside, kaempferol-3-O-glucoside, Niazicin-A, Niazimin-A, and Niaziminin-B	Alleviation of vascular dysfunction and oxidative stress, blunted adrenergic-mediated vasoconstriction, promoted endothelium-dependent vasorelaxation; inhibition of angiotensin-converting enzyme	*In vivo* assay in L-NAME-treated rats; *in vitro* angiotensin-converting enzyme inhibitory assay; *in silico* molecular interaction	[79–81]
*Moringa stenopetala (Baker f.)*	Moringaceae	Leaves	Alkaloids, flavonoids, and saponins	Inhibition of carbonyl anhydrase	*In vivo* assay on mice	[82]
*Musa sapientum*	Musaceae	Fruit peel	(±)−7, 8-Dihydroxy-3-methyl-isochromanone-4 (polyphenol)	Reduction of oxidative stress and increase in NO by activation of pathway PI3K/Akt/eNOS	*In vivo* assay in spontaneously hypertensive rats	[83]
*Nardostachys jatamansi*	Caprifoliaceae	Rhizome	Jatamansone, calarene, spirojatamol, aristolone, valencene and patchouli alcohol, *α*-pinene, and *β*-maaliene	Inhibition of angiotensin-converting enzyme	*In vitro* angiotensin-converting enzyme inhibitory assay	[84]
*Onopordum acanthium*	Asteraceae	Seed	(E)−1-oxo-3, 4-dihydro-1-H-isochromen-7-yl-3-(3, 4-dihydroxyphenyl) acrylate	Inhibition of angiotensin-converting enzyme	Molecular interaction *in silico in vitro* assays	[85]
*Orthosiphon stamineus*	Lamiaceae	Leaves	No data	Modulation of *α*1-adrenergic receptors and AT1 and increase in levels of NO	A parallel-group, randomized, placebo-controlled study in humans; rings of aorta of spontaneously hypertensive rats	[86]
*Panax notoginseng*	Araliaceae.	Root	Ginsenoside Rg1 and Rb1	NO/sGC/cGMP pathway and *β*2-adrenergic receptors	*Ex vivo* rat assays in isolated tissue preparations (aortic ring model)	[87]
*Peperomia pellucida*	Piperaceae	Leaves	2, 3, 5-trimethoxy-9-(12, 14, 15-trimethoxybenzyl)-1H-indene and pellucidin A	Inhibition of angiotensin-converting enzyme	*In vitro* angiotensin-converting enzyme inhibitory assay	[88]
*Phaseolus vulgaris*	Fabaceae	Seed	Catechins, flavonoids, and *γ*-aminobutyric acid (GABA)	Inhibition of angiotensin-converting enzyme and modulation of pressure via GABA.	*In vitro* assays	[89]
*Phoenix dactylifera*	Arecaceae	Fruits	Squalene, lauric acid, palmitic acid, caprate, stearate, vitamin E, *β*-sitosterol, phytol, linolenic acid, isosorbide, coumarins, and taurine	Inhibition of angiotensin-converting enzyme	*In vitro* enzyme inhibition assays	[90]
*Piper nigrum*	Piperaceae	Seed	Piperine (alkaloid)	Reduces oxidative stress	*In vivo* assay in rats with hypertension caused by obesity induced by a lipid-rich diet	[91]
*Prunus persica*	Rosaceae	Aerial parts	Amygdalin, cyanogenic glycosides, prunasin, caffeic acid, chlorogenic acid, kaempferol, p-coumaric acid, prussic acid, quercetin, quercitrin, quinic acid, tannin, and ursolic acid	NO-sGC-cGMP, vascular prostacyclin, and muscarinic receptor transduction pathway	*Ex vivo* rat assay in isolated tissue preparations (aortic ring model)	[92]
*Rauvolfia serpentina*	Apocynaceae	Roots	Reserpine, ajmalicine, serpentinine, ajmalimine, ajmaline, rescinnami- dine, rescinnamine, reserpiline, serpentine, indobidine, yohimbine, and deserpidine	Protecting the liver and renal architectures	*In vivo* assay in rats with hypertension induced by high salt diet	[93]
*Rubus rosifolius*	Rosaceae	Leaves	Escauphic acid, flavonoids, and triterpenes	Diuretic effect	*In vivo* assay in hypertensive male rats	[94]
*Salvia miltiorrhiza*	Lamiaceae	Root	Lithospermic acid B	Inhibition of angiotensin-converting enzyme	*Ex vivo* assays for vasodilation in rat aortic rings	[95]
		Root	*Tanshinoato* of *magnesium B*	Increase in NO levels	*In vivo* assay in rats with phenylephrine-induced hypertension	[96]
*Salvia scutellarioides*	Lamiaceae	Aerial parts	Alkaloids, triterpenes, lignans, and flavonoids	Vasodilation, which activates compensatory physiological responses such as the renin-angiotensin-aldosterone system, and increase in concentrations of epinephrine and vasopressin	*In vivo* assay in L-NAME-treated rats	[97]
*Sargassum siliquastrum* ^*∗∗*^	Sargassaceae	Entire organism	*Sargachromenol D*	Induced depolarization	*In vivo* assay in rat basilar arteries	[98]
*Sceletium tortuosum*	Mesembryathemaceae	Leaves	Mesembrine (alkaloid)	Inhibition of aldosterone synthesis	*In vitro* assay on the culture of human adrenocortical carcinoma cells	[99]
*Solanum donianum*	Solanaceae	Leaves	Unreported	Inhibition of angiotensin-converting enzyme	*In vitro* angiotensin-converting enzyme inhibitory assay	[100]
*Spirulina maxima* ^*∗∗*^	Cyanophyceae	It has no true tissues	Phycocyanin	Increases transcription of the enzyme eNOS	Cohort study with humans	[101]
*Taraxacum officinale*	Asteraceae	Leaves and root	Saponins, alkaloids, phenols, flavonoids, tannins, and glycosides	Increase in NO levels by eNOS (inducible NO synthase)	*In vivo* assay in L-NAME-treated rats and with spontaneously hypertensive rats	[102]
*Taxus chinensis var. mairei*	Taxaceae Gray	Leaves	Palmitic acid, 9-octan-dienate of hexadecanil, and octan-3-ol	Reduction of the level of angiotensin II and increase in NO levels	*In vivo* assays with mice with hypertension by chronic nitric oxide inhibition and *in vitro* assays	[103]
*Terminalia superba*	Combretaceae	Stem bark	Saponins, glycosides, flavonoids, and chalcones	Reduction of oxidative stress	*In vivo* assays with mice with glucose-induced hypertension (GHR); *ex vivo* assays that evaluate the cellular redox state	[104]
*Ulmus wallichiana*	Ulmaceae	Stem bark	Flavonoids analogous to quercetin	Modulation of the renin-angiotensin-aldosterone system and stimulation of NO/cGMP pathway	*In vivo* assay in spontaneously hypertensive rats and assays in rats with salt and mineralocorticoid-induced hypertension, and with rats with chronic inhibition of nitric oxide	[105]
*Urtica dioica*	Urticaceae	Aerial parts	No data	An important bradycardia, which is independent of cholinergic and 1-adrenergic receptors	*Ex vivo* assays in isolated Langendorff perfused rat heart and vasodilation in rat aortic rings	[42]
*Vaccinium virgatum*	Ericaceae	Fruit	Anthocyanins and polyphenols	Stimulation of NO/cGMP pathway	A double-blind, randomized, placebo-controlled study in humans	[106]
*Vaccinium corymbosum*	Ericaceae	Fruit	Anthocyanins and polyphenols	Stimulation of NO/cGMP pathway	A double-blind, randomized, placebo-controlled study in humans	[106]
*Vitex cienkowskii*	Lamiaceae	Stem bark	Tetra-acetyl jugasterone C	Stimulation of NO/cGMP pathway and blockade of transmembrane calcium influx	*Ex vivo* tests on preparations of tissues isolated from rats	[107]
*Zea mays*	Poaceae	Seed	Corn peptide	Inhibition of angiotensin-converting enzyme	*In vivo* assay in spontaneously hypertensive rats and *in vitro* assays	[108]

^*∗*^Fungus species and ^*∗∗*^species of seaweed.
